The article "Advancing Perioperative Neurocognitive Health: A Critical Review of Predictive Tools, Diagnostic Methods, and Interventional Strategies" was retracted in 2025. Reasons: unreliable results or conclusions; concerns about the citations.

# Advancing Perioperative Neurocognitive Health: A Critical Review of Predictive Tools, Diagnostic Methods, and Interventional Strategies

**DOI:** 10.7759/cureus.59436

**Published:** 2024-05-01

**Authors:** Swetha Lakshminarayanan, Mohazin Aboobacker, Anureet Brar, Mathew Parackal Manoj, Mostafa Mohamed Elsaid Ismail Elnimer, Aamuktha Marepalli, Krutarth Jay Shukla, Muhammad Sheraz Yousaf, Ahsen Taqveem, Muhammad Junaid Hassan

**Affiliations:** 1 General Surgery, Sri Ramachandra Institute of Higher Education and Research, Chennai, IND; 2 Neurosurgery, Jubilee Mission Medical College and Research Institute, Thrissur, IND; 3 Neurology, Sri Guru Ramdas Institute of Medical Sciences and Research, Amritsar, IND; 4 General Surgery, Government Medical College Kottayam, Kottayam, IND; 5 Gastroenterology, Kafr Elsheikh Liver Research Center, Kafr El-Sheikh, EGY; 6 Medicine, Sri Venkateswara Institute of Medical Sciences, Tirupati, IND; 7 Medicine, Gujarat Cancer Society Medical College Hospital and Research Centre, Ahmedabad, IND; 8 Medicine, Faisalabad Medical University, Faisalabad, PAK; 9 Microbiology, Government College University Faisalabad, Faisalabad, PAK; 10 Internal Medicine, Faisalabad Medical University, Faisalabad, PAK

**Keywords:** neurocognitive disorders, geriatric surgical population, perioperative cognitive impairment, risk mitigation strategies, neurocognitive rehabilitation, cognitive assessment, general anesthesia, perioperative neurocognitive disorder

## Abstract

Perioperative neurocognitive disorders (PNDs) affect a large percentage of people who undergo surgeries that need general anesthesia. There is an increased risk of death and a major disruption to postoperative self-care as a result of this. This study compiles all the relevant materials that the authors have found to investigate postnatal depression and its causes, as well as the methods used to determine the probability and severity of PNDs and how to reduce their risk before surgery. Postnatal depression can have many causes, and this text explores some of them. These include a history of alcohol or opiate use, immunological dysregulation, advanced age, educational background, infections, neurocognitive impairment, and pre-existing chronic inflammatory disorders. It also delves into various methods used to gauge the likelihood and severity of postpartum depression. The following assessment tools were covered: the Clock Drawing Test, Domain-Specific Tests, the Mini-Mental State Examination, and the Montreal Cognitive Assessment. In addition to biochemical markers, neuroimaging techniques play an important role in diagnosis. The Frailty Fried assessment, which measures inertia, sluggishness, lack of physical activity, fatigue, and unintentional weight loss, is a key prognostic sign that is highlighted. There is strong evidence that the index, which is derived from these five characteristics, may accurately predict the likelihood of PNDs. Risk mitigation strategies are also covered in this research. Preoperative brain plasticity-based therapies, such as physical exercise and intensive cognitive training, can significantly reduce the incidence and severity of postoperative neurocognitive disorders. A peripheral nerve block, monitoring cerebral oxygen saturation, dexmedetomidine, and a reduction in anesthesia depth are all ways to improve anesthetic procedures. Methods that lower blood pressure should be avoided, the body temperature should be kept down during surgery, or the time without liquids should be lengthened; all of these raise the risk of postoperative nausea and vomiting and make it worse. Potential approaches include a Mediterranean diet, physical activity, cognitive stimulation, smoking cessation, alcohol reduction, avoidance of anticholinergic medications, and non-steroidal anti-inflammatory drug stewardship, although there is no definitive evidence for successful postoperative neurocognitive rehabilitation procedures. More standardized diagnostic criteria, evaluation methods, and PND classification are urgently needed, according to this study. Different cases of PNDs are characterized by different combinations of tests, cutoff values, and methods because there is a broad variety of diagnostic tests used to make the diagnosis. Until now, PNDs and pre-existing neurocognitive disorders have been diagnosed using the Diagnostic and Statistical Manual of Mental Disorders (DSM-V). With an aging population comes an increase in the occurrence and prevalence of PNDs, which calls for a specific way to classify and describe the condition.

## Introduction and background

Cognitive decline occurs in 10-40% of patients before, during, or after surgery, and the number of procedures performed on older adults has been on the rise [1]. Neurocognitive impairment is seen in around 21.2-28% of people in this age range and it is similar to the postoperative neurocognitive abnormalities seen in surgical patients. Neurocognitive impairments following surgery should be clearly distinguished from those resulting from pre-existing diseases such as moderate cognitive impairment, dementia, or Alzheimer's disease [2]. Many people experience various forms of cognitive impairments leading up to, during, and after surgery; these are collectively known as perioperative neurocognitive disorders. All preoperative neurocognitive impairments, acute neurocognitive abnormalities (like postoperative delirium), and cognitive declines occur within 30 days and 12 months after surgery [3]. A significant decrease in quality of life and independence may result from perioperative neurocognitive disorder (PND's) negative impacts on learning, memory, focus, attention, and psychomotor function. According to recent research, there is an increased death rate among persons whose neurocognitive impairment persists for at least three months following treatment.

A study found that no matter the age group, no more than 4.3% of patients experienced postoperative delirium symptoms after surgery. The study indicated that among those older than 70 years old, 10.5% had it [4]. There was a 9.9% incidence of delayed postoperative cognitive recovery at 99 days and a 25.8% incidence at seven days, according to another study. Postpartum depression is more common in older adults, those with less education, those who smoke, those who use certain drugs, and those who are genetically predisposed to the disorder, according to research. Postnatal depression is a serious mental health issue, and this study intends to investigate its causes, symptoms, diagnostic tools, and potential solutions [5].

## Review

Risk factors for PNDs in perioperative settings

Multiple factors interact to cause perioperative noncommunicable diseases. Triggering variables and predisposing factors are two ways to classify the complex etiology of PNDs [6]. According to research, one controllable element that can impact the onset of postpartum depression is the choices people make on a daily basis. Many diseases that affect the elderly, including infections, autoimmune disorders, and chronic inflammatory diseases, are thought to be exacerbated by inflammation. Being above the age of 60 is known to increase the likelihood of developing postnatal depression [7]. Clinical trials have revealed several key risk factors for PND, including advanced age, a history of alcohol or opiate misuse, a lack of education, a history of severe surgical procedures, the use of anticholinergic medication, and pre-existing cognitive impairment [8]. Among the many postoperative neurocognitive disorders (NCDs), delirium is more commonly associated with advanced age and prior cognitive impairment. In adults, delirium following surgery occurs between 2.5 and 4.5 percent of the time. In patients 60 and up, the risk of postoperative delirium rises from 12.0% to 23.8%. Immune dysregulation, characterized by increased blood levels of pro-inflammatory cytokines, is a hallmark of aging. Dementia is significantly connected with PNDs, which include acute postoperative delirium and persistent postoperative cognitive impairment. PNDs are age-related neurological illnesses [9,10]. A large percentage of patients 65 and older had moderate to severe neurocognitive impairment before surgery. Since these people are more likely to experience postoperative delirium, chronic neurocognitive impairment, or later-stage dementia, identifying them is crucial. Testing coronavirus disease 2019 (COVID-19) for the possibility of acute and chronic neurological problems is crucial since SARS-CoV-2 is more invasive in the CNS than other coronaviruses. Changes in the epidemiological features of numerous diseases have been triggered by the COVID-19 pandemic. The blood-brain barrier can be broken after surgery or anesthesia, allowing innate immune molecules from the outside world to enter the hippocampus. According to certain sources, SARS-CoV-2 may speed up this process [11,12]. Postnatal depression and COVID-19 are both linked to mitochondrial malfunction, according to mounting evidence. By binding to the ACE-2 receptor, SARS-CoV-2 can influence mitochondria, causing them to fuse and overproduce reactive oxygen species. Mitochondrial DNA is damaged and oxidative stress in the CNS is accelerated in this process. Whether or not delirium develops during an operation depends on its unique features and scope. Patients undergoing heart surgery (15.3-23.4%), hip fracture surgery (16.9%), emergency surgery (22.7-26%), and intensive care unit admission following surgery (24.4%) had higher rates of delirium, according to other studies [13].

All forms of systemic inflammation following surgery have a common denominator: the inflammatory response that the surgical procedure itself causes. The fact that the brain is already inflamed or showing signs of degeneration could be the reason why it is more vulnerable to a systemic inflammatory response. Still, it's possible that the patient won't notice or acknowledge this. In order to reduce the risk of postoperative delirium and postoperative NCDs, it is important to rule out the possibility of dementias like Alzheimer's while planning surgery [14]. Postpartum depression is more common among those with less education. Conversely, it is possible to view a higher degree of schooling as a sign of cognitive reserve, which aids in protecting against PNDs. Postpartum depression is more likely in women who have a history of sleep disorders, who drink to excess, who take multiple medications or psychotropic drugs, and who have certain medical conditions like diabetes, severe vascular disease, frailty, or neuronal damage from a stroke or traumatic brain injury (Figure 1) [15,16].

**Figure 1:** The role of astrocytes in neuroinflammation and the blood–brain barrier. IL-1α: interleukin-1α; TNF-α: tumor necrosis factor α; C1q: component 1q; C3: component C3; Aβ: β-amyloid; Cx43: gap junctions-connexin 43; BDNF: brain-derived neurotrophic factor. Reproduced under the terms and conditions of the Creative Commons Attribution (CC BY) license from ref [17]. Copyright © 2022 by the authors. Licensee MDPI, Basel, Switzerland.

Assessing methods for the common evaluation of cognitive decline during surgery

The Mini-Mental State Examination is among the most widely used tests of cognitive ability. The MMSE (Mini-Mental State Examination) showed sensitivity and specificity in detecting dementia that were intermediate, according to a meta-analysis of 34 trials. The sensitivity ranged from 77% to 83% and the specificity from 87% to 91%, depending on the clinical scenario. On the other hand, its specificity was just 65% and sensitivity was 63% when it came to diagnosing mild neurocognitive dysfunction [18]. For moderate neurocognitive dysfunction, a separate meta-analysis indicated similar sensitivity (62%). In order to assess a broader range of cognitive abilities, researchers developed a new version of the MMSE called the modified MMSE (or 3 multiple sclerosis) [19]. When it comes to detecting mild NCDs, the modified MMSE is 84% more sensitive than the standard MMSE, which is 58% sensitive. On the other hand, the MMSE has been underutilized in both academic and clinical settings.

Many people opt to take the Montreal Cognitive Assessment (MoCA) instead of the Mini-Mental State Examination. When compared to the MMSE and the modified MMSE, its sensitivity for identifying mild NCDs is 90%. Although the difference is not very large, a recent meta-analysis demonstrated that MoCA is superior to MMSE in diagnosing moderate NCDs. MoCA had a sensitivity of 81% and specificity of 74%, based on 24 studies and a sample size of 4,095, while MMSE had a sensitivity of 66% and specificity of 74%, based on 46 studies and a sample size of 17,749. Compared to MMSE (81%), MMMSE (86%), and MoCA (91%), a meta-analysis showed that MoCA was superior in detecting frank dementia [20].

Additionally, the Consortium to Establish a Registry for Alzheimer's Disease (CERAD) neuropsychological assessment battery and the Addenbrooke's Cognitive Examination-Revised were both included in the meta-analysis of comprehensive cognitive tests. Despite their relative obscurity, both tests are just as sensitive (82% for both tests) and specific (78% and 76% respectively) as MoCA in identifying mild NCDs. When compared to the MoCA test, a newer version of the Addenbrooke's Cognitive Examination-Revised (ACE-R), called ACE-III, has shown better sensitivity (97% vs. 91% specificity) for identifying moderate neurocognitive dysfunction. Unfortunately, there is a lack of sufficient evidence in this particular patient population to fully confirm the use of e7 in perioperative settings. In addition, tests that are both shorter and less complicated have shown promise in detecting cognitive decline. The Clock-Drawing Test (CDT) e8-e10 is one of the tests that are specified. Memory decline is often a significant element in early cognitive impairment, and the CDT does not include a memory evaluation, so it is not very useful for cognitive screening [21,22]. 

In comparison to the MMSE (81% sensitivity and 89% specificity), the Mini-Cognitive Assessment (Mini-Cog) test (which consists of a clock-drawing task and a three-item memory recall test) showed a higher sensitivity (91%) and specificity (86%). Its results were comparable to those of the MoCA (91% sensitivity and 81% specificity) and the ACE-R (92% specificity and 89% sensitivity). There isn't enough proof that the Mini-Cog test can identify moderate neurocognitive dysfunction, yet it's a good tool for dementia diagnosis. On the other hand, mild NCDs can be identified using the Quick Mild Cognitive Impairment test. This has been supplied by the user. The Qmci test outperformed the MMSE and MoCA in differentiating moderate NCD from healthy controls, as shown in a comprehensive evaluation. In comparison to the MMSE (61% sensitivity, 67% specificity) and the MoCA (79% specificity), the Qmci test was the most sensitive and specific (82%) of the three.

In addition to the more traditional "pen and paper" cognitive tests, computer-based exams have also been developed as a consequence of technological progress. In many contexts, including those following surgery, the Cogstate Brief Battery (CBB) is an effective cognitive assessment tool. It can detect mild NCDs in people of all ages, even those who don't have much experience with computers. The sensitivity (80%) and specificity (85%) of CBB in detecting moderate NCDs are similar to those of MoCA; there are two major downsides to keep in mind. First of all, it's proprietary, which means that information belongs to a particular corporation and could cost more to use. Secondly, because the evaluation is done online, there can be worries about personal data security [23].

Matching tools to disease: improving clinical care and patient outcomes

Doctors need to be familiar with a variety of cognitive screening tools for different surgical scenarios, as there is no one-size-fits-all instrument. This variety helps in detecting and managing cognitive impairments during perioperative procedures [23]. In order to assess patients' cognitive capacities before and after surgery, optimal cognitive screening entails administering tests both before and after the operation. Because people are different, it could be hard to draw broad conclusions from data collected from normative populations. However, it may still be beneficial to do preoperative screening on its own when assessing risk (i.e., to identify preexisting cognitive impairment, which may foretell postoperative cognitive issues). If preoperative testing is not possible, postoperative follow-ups may nevertheless help afflicted patients find the right therapy. Thus, we will address the unique concerns of each perioperative scenario in the section that follows. For precise monitoring of cognitive trajectories throughout the perioperative period, it is essential to choose a single screening tool that is appropriate for both preoperative and postoperative screening. The reason being, it's not easy to compare scores from various tools. Below, we will go over a few of these types of tests [24].

Preoperative cognitive screening

In busy settings like emergency departments and preoperative clinics, where patients need examination, efficient screening is desirable. Furthermore, preoperative screening should be conducted for all senior patients, irrespective of subjective symptoms or prior suspicion of cognitive impairment, since a mild NCD is often asymptomatic and remains undetected. Therefore, this is not the best setting for tests that take longer than a few minutes to finish. It is not practical to employ preoperative screening tests like MMSE and CDT, which have low sensitivity for identifying mild neurocognitive problems, for this purpose. The reason being, any history of cognitive impairment, no matter how modest, is a strong predictor of postoperative cognitive and noncognitive complications [24].

When compared to other paper-based screening tests, such as the MoCA and the MMSE, the Qmci stands out for its greater sensitivity and specificity, in addition to its quick and easy administration. However, Quick Mild Cognitive Impairment screen (Qmci) has not been used in perioperative contexts prior to this. However, because of its rapid administration and precise dementia detection capabilities, the Mini-Cog test has seen significant application in preoperative screening. Its limited use stems from the fact that it fails to identify mild NCDs. Hence, MoCA may be a better screening approach than other options, even if it takes more time to administer. It has also been validated more thoroughly and has equivalent sensitivity. Individuals detected by early screening may be directed to undergo more extensive testing in order to get a definitive diagnosis, regardless of the test used.

Patients might be given the option to take cognitive tests at home before their planned session, rather than having to go to a preparatory clinic. Sensitivity to mild neurocognitive impairments and the ability to remotely deliver the medication may take precedence in this setting over administration time. Among computerized tests, the Computer-Administered Montreal Cognitive Assessment (CAMCI) stands out for its exceptional sensitivity (86%) in identifying mild NCDs. Furthermore, it is self-administered in older individuals, but its particular efficacy in the preoperative setting is still up for debate [25].

In-hospital cognitive assessment after surgery

The rate of administration is much lower in the postoperative period compared to the preoperative clinic. Here, test-retest reliability is second only to the absolute need for accurate detection of cognitive change. This is because a patient's cognitive trajectory may be assessed by periodic postoperative testing. With a good test-retest reliability (r = 0.88-0.92)10 and a significant ability to properly detect mild neurocognitive abnormalities, MoCA is an appropriate option among traditional tests. It has also been tested and shown to be safe for use throughout the time leading up to surgery [26]. Although the sensitivity and specificity of the ACE-R and CERAD tests are similar, the results of the MoCA study are more applicable since they are based on a bigger sample and a broader range of clinical settings. In settings where computers and tablets are readily available, CBB and CAMCI work well. Whereas traditional "pen and paper" exams are prone to bias, errors, and learning effects, these alternatives are superior. The Cognitive Assessment Battery's (CBB) principal goal was to confine the assessment to executive functioning, attention, and memory in order to minimize the influence of practice effects. The perioperative context is just as valid as the other, with the same amount of time commitment required and equivalent sensitivity and specificity to MoCA. Although the CAMCI test is more time-consuming and has not been shown to be reliable during the perioperative period, it has demonstrated higher sensitivity (86% and 94%, respectively) in identifying mild NCDs in one study. This contradicts the findings of a previous meta-analysis that showed the MoCA test to be 74% specific and 81% sensitive [27].

Postoperative cognitive change after hospital discharge

After a patient leaves the hospital, remote administration is a great way to track their cognitive growth. This makes cognitive testing more accessible and lessens the need for patients, particularly those in remote or rural locations, to make many trips to the hospital. Computerized tests like CBB and CAMCI could prove to be the best in this regard. If a patient's test results show signs of cognitive loss, their primary care physician or a specialist may recommend more testing, such as a more comprehensive neuropsychological or cognitive examination. Other factors, such as patients' subjective reports of memory issues and the impact these problems have on their everyday lives, should be considered before reaching a definitive diagnosis. Still, it could be useful to have a screening tool that is both objective and proven (Figure 2) [28].

**Figure 2:** (A) Five main pathogenic hypotheses that have been proposed to explain the emergence and progression of POD, which is defined by disruptions in attention, consciousness, and cognition. The activation of TLR4 in macrophages and microglia is promoted by S100A8, a prominent member of DAMPs. (B) This activation leads to an increase in the expression of TNF-α, which binds to TNFR on endothelial cells and triggers their necroptosis. This process undermines the integrity of the BBB and increases its permeability. POD: Postoperative delirium; TLR4: toll-like receptor 4; S100A8: S100 calcium-binding protein A8; DAMPs: damage-associated molecular patterns; TNF-α: tumor necrosis factor α; TNFR: tumor necrosis factor receptor; BBB: blood-brain barrier. Reproduced under the terms and conditions of the Creative Commons Attribution (CC BY) license from ref [29]. Copyright © 2022 by the authors. Licensee MDPI, Basel, Switzerland.

Diagnosis of NCDs

Diagnosis of Delirium

In accordance with the DSM-5 terminology, the most recent consensus acknowledges postoperative delirium as a separate category. Symptoms usually start appearing soon after surgery [30]. A case of postoperative delirium meets the diagnostic criteria as out by the DSM-5 when it develops during a hospital stay, continues for at least seven days after surgery or until discharge, and is considered a newly acquired disorder [31]. Delirium that develops after discharge is no longer considered "postoperative" unless it persists throughout the hospital stay, beginning during the postoperative phase. When diagnosing delirium, it is crucial to differentiate between two types: developing delirium and postoperative delirium. Patients could experience an episode of emergent delirium while under general anesthesia or soon after waking up. Within a few hours or minutes, it usually disappears. However, postoperative delirium often occurs within the first 24 to 72 hours after surgery and normally resolves itself within a few days. The postanesthesia care unit is the primary location for observing and evaluating patients with emergent delirium, whereas the primary location for monitoring patients with postoperative delirium begins the day after surgery (Figure 3) [32,33].

**Figure 3:** Recent papers published on Pubmed® regarding postoperative delirium in the last five years. Reproduced under the terms and conditions of the Creative Commons Attribution (CC BY) license from ref [34]. Copyright © 2022 by the authors. Licensee MDPI, Basel, Switzerland.

For the purpose of diagnosing postoperative delirium, the DSM-5 is the gold standard. Users outside of the mental health field see DSM-5 as having little practical application to their work. The development and validation of more than 20 diagnostic tools have greatly improved the process of delirium diagnosis [35,36]. The following are examples of frequently used screening tools for evaluating confusion: Confusion Assessment Method, the Confusion Assessment Method for the Intensive Care Unit, the Brief Confusion Assessment Method, the Intensive Care Delirium Screening Checklist, and the 4A's Test. One hundred and eight different delirium assessment tools have been tested and proven to work. To gauge the severity of delirium, three main instruments are used: Memory Delirium Assessment Scale, the Delirium Rating Scale-Revised-98, and the Confusion Assessment Method-degree [37].

Diagnosis of delayed neurocognitive recovery and postoperative cognitive dysfunction

The standard for determining NCDs is a "small or substantial decrease in performance from the prior level in one or more cognitive domains (complex attention, executive function, learning and memory, language, perceptual-motor, or social cognition)." The traditional method for assessing the performance of various cognitive areas involves administering a battery of neuropsychological tests. The three most often administered individual neuropsychological tests are the digit span test (including both forward and backward subtests), the trail-making test part A, and the digit symbol substitution test [38,39]. The Montreal Cognitive Assessment, the Addenbrooke's Cognitive Exam, and the Quick MCI Screen are three short tools that are currently being used to identify mild cognitive impairment [40-43].

According to the DSM-5, a moderate NCD is described as a decrease of 1-2 standard deviations (for normally distributed test results) or between the 3rd and 16th percentile (for non-normally distributed test results). Conversely, a drastic drop below the third percentile (in a non-normal distribution) or more than two standard deviations (in a normal distribution) is indicative of a significant NCD. Having normal or baseline data is essential for using the aforementioned cut-points to determine the degree of cognitive changes. In studies with both a baseline and a control group, the z-score is often computed. The z-score is determined by subtracting the mean practice effect from the difference between each test's results before and after surgery. The control group's standard deviation is then used to split this result. After adding together all of a patient's test z-scores and standardizing them using the control group's normal deviations, we get their composite z-score. Individual test z-scores or composite z-scores equal to or less than -1.96 indicate cognitive deterioration [44].

A totally objective decline in cognitive function is required for the diagnosis of postoperative cognitive dysfunction (POCD), which is currently reserved for research contexts [44]. Evidence of cognitive decline is required for a diagnosis of NCDs, in contrast to POCD, which just requires the presence of cognitive problems and an evaluation of daily functioning. People, informants, or medical professionals may report cognitive problems. A thorough assessment of cognitive difficulties should be carried out via the process of recording a patient's history both before and after surgery. A good device may be used to evaluate daily activity and identify slight differences. Someone close to the person or the person themself might potentially report it. A mild neurocognitive disease requires maintaining everyday functioning to a greater or lesser extent than a severe NCD. Cognitive symptoms and daily activity evaluation during hospitalization and after discharge might be problematic due to pharmacological and surgical interventions. Accordingly, the Nomenclature Consensus Working Group 1 proposes the term "delayed neurocognitive recovery" to describe the "NCD" condition that occurs in the first 30 days after surgery. From that point on, until 12 months after surgery, the phrase "postoperative mild/major NCD" should be used. A diagnosis must be made during the 12-month timeframe in order for the term "postoperative" to be appropriate [45,46].

## Conclusions

In conclusion, PNDs represent a significant challenge in the care of surgical patients, particularly among the elderly and those with pre-existing risk factors such as cognitive impairments, substance use, and chronic inflammatory conditions. The investigation into PNDs underscores the complexity of their etiology, highlighting the multifactorial nature of their risk factors and the critical role of early identification and intervention. The review of diagnostic tools, including the Clock Drawing Test, Mini-Mental State Examination, and Montreal Cognitive Assessment, underscores the importance of accurate and early diagnosis in managing PNDs effectively. Furthermore, the exploration of risk mitigation strategies emphasizes the potential of preoperative interventions, such as cognitive training, alongside intraoperative measures like monitoring cerebral oxygen saturation and maintaining optimal anesthesia depth, to significantly reduce the incidence and impact of PNDs. The collective insights from this review call for a multidisciplinary approach to perioperative care, integrating tailored risk assessment, vigilant monitoring, and targeted interventions to minimize the cognitive sequelae of surgery and enhance patient recovery and quality of life.

## References

[1] Hasan TF, Kelley RE, Cornett EM, Urman RD, Kaye AD (2020). Cognitive impairment assessment and interventions to optimize surgical patient outcomes. Best Pract Res Clin Anaesthesiol.

[2] Deiner S, Liu X, Lin HM (2021). Does postoperative cognitive decline result in new disability after surgery?. Ann Surg.

[3] Spies C, Knaak C, Lachmann G, Heinrich M (2023). Mission - Innovation : Telematics, eHealth and High-Definition Medicine in Patient-Centered Acute Medicine. https://levana.leopoldina.org/receive/leopoldina_mods_00361.

[4] Lammers-Lietz F, Borchers F, Feinkohl I (2024). An exploratory research report on brain mineralization in postoperative delirium and cognitive decline. Eur J Neurosci.

[5] Gedzyk-Nieman SA (2021). Postpartum and paternal postnatal depression: identification, risks, and resources. Nurs Clin North Am.

[6] Kanyongo W, Ezugwu AE (2023). Feature selection and importance of predictors of non-communicable diseases medication adherence from machine learning research perspectives. Informatics in Medicine Unlocked.

[7] Hoseini-Tavassol Z, Ejtahed HS, Larijani B, Hasani-Ranjbar S (2023). Trimethylamine N-oxide as a potential risk factor for non-communicable diseases: a systematic review. Endocr Metab Immune Disord Drug Targets.

[8] Ma J, Wang F, Wang J, Wang P, Dou X, Yao S, Lin Y (2023). The effect of low-dose esketamine on postoperative neurocognitive dysfunction in elderly patients undergoing general anesthesia for gastrointestinal tumors: a randomized controlled trial. Drug Des Devel Ther.

[9] McKnight R, Price J, Geddes J (2019). 26 Delirium, dementia, and other cognitive disorders. Oxford Academic.

[10] Evered LA, Goldstein PA (2021). Reducing perioperative neurocognitive disorders (PND) through depth of anesthesia monitoring: a critical review. Int J Gen Med.

[11] Tang X, Yv H, Wang F (2022). The relationship between suboptimal social networks and postoperative delirium: the PNDABLE study. Front Aging Neurosci.

[12] Liu F, Lin X, Lin Y, Deng X, Dong R, Wang B, Bi Y (2022). Subjective cognitive decline may mediate the occurrence of postoperative delirium by P-tau undergoing total hip replacement: the PNDABLE study. Front Aging Neurosci.

[13] Bhattacharya S, Basu P, Poddar S (2020). Changing epidemiology of SARS-CoV in the context of COVID-19 pandemic. J Prev Med Hyg.

[14] Dilmen OK, Meco BC, Evered LA, Radtke FM (2024). Postoperative neurocognitive disorders: a clinical guide. J Clin Anesth.

[15] Albanese AM, Ramazani N, Greene N, Bruse L (2022). Review of postoperative delirium in geriatric patients after hip fracture treatment. Geriatr Orthop Surg Rehabil.

[16] Chen X, Li L, Yang L, Li A, Wu M, Yu D (2023). A Randomised Trial: BIS-Guided Anesthesia Decreases The Incidence of Delayed Neurocognitive Recovery And Postoperative Neurocognitive Disorder But Not Postoperative Delirium. https://www.researchsquare.com/article/rs-505070/v2.

[17] Cao Y, Lin X, Liu X, Yu K, Miao H, Li T (2022). The role of astrocytes in the mechanism of perioperative neurocognitive disorders. Brain Sci.

[18] Zhang B, Li D, Liu Y, Wang J, Xiao Q (2021). Virtual reality for limb motor function, balance, gait, cognition and daily function of stroke patients: a systematic review and meta-analysis. J Adv Nurs.

[19] Alonso RN, Eizaguirre MB, Silva B (2020). Brain function assessment of patients with multiple sclerosis in the expanded disability status scale: a proposal for modification. Int J MS Care.

[20] Rost NS, Brodtmann A, Pase MP (2022). Post-stroke cognitive impairment and dementia. Circ Res.

[21] Bello-Lepe S, Alonso-Sánchez MF, Ortega A, Gaete M, Veliz M, Lira J, Perez Salas CP (2020). Montreal cognitive assessment as screening measure for mild and major neurocognitive disorder in a Chilean population. Dement Geriatr Cogn Dis Extra.

[22] Limpawattana P, Manjavong M (2021). The Mini-Cog, clock drawing test, and three-item recall test: rapid cognitive screening tools with comparable performance in detecting mild NCD in older patients. Geriatrics (Basel).

[23] De Roeck EE, De Deyn PP, Dierckx E, Engelborghs S (2019). Brief cognitive screening instruments for early detection of Alzheimer's disease: a systematic review. Alzheimers Res Ther.

[24] Decker J, Kaloostian CL, Gurvich T (2020). Beyond cognitive screening: establishing an interprofessional perioperative brain health initiative. J Am Geriatr Soc.

[25] Mattke S, Batie D, Chodosh J (2023). Expanding the use of brief cognitive assessments to detect suspected early-stage cognitive impairment in primary care. Alzheimers Dement.

[26] Katz MJ, Wang C, Nester CO (2021). T-MoCA: a valid phone screen for cognitive impairment in diverse community samples. Alzheimers Dement (Amst).

[27] O'Gara BP, Mueller A, Gasangwa DV (2020). Prevention of early postoperative decline: a randomized, controlled feasibility trial of perioperative cognitive training. Anesth Analg.

[28] Bourgeois JA, Giroux C (2024). Consultation-liaison psychiatry. Geriatric Psychiatry: A Case-Based Textbook.

[29] Xu Y, Ma Q, Du H, Yang C, Lin G (2022). Postoperative delirium in neurosurgical patients: recent insights into the pathogenesis. Brain Sci.

[30] Evered L, Silbert B, Knopman DS (2018). Recommendations for the nomenclature of cognitive change associated with anaesthesia and surgery—2018. Anesthesiology.

[31] Herrman H, Patel V, Kieling C (2022). Time for united action on depression: a Lancet-World Psychiatric Association Commission. Lancet.

[32] Zhang Y, He ST, Nie B, Li XY, Wang DX (2020). Emergence delirium is associated with increased postoperative delirium in elderly: a prospective observational study. J Anesth.

[33] Su X, Meng ZT, Wu XH (2016). Dexmedetomidine for prevention of delirium in elderly patients after non-cardiac surgery: a randomised, double-blind, placebo-controlled trial. Lancet.

[34] Melegari G, Gaspari A, Gualdi E (2022). Delirium in older adults: what a surgeon needs to know. Surgeries.

[35] Oh ES, Fong TG, Hshieh TT, Inouye SK (2017). Delirium in older persons: advances in diagnosis and treatment. JAMA.

[36] Marcantonio ER (2017). Delirium in hospitalized older adults. N Engl J Med.

[37] Wilson JE, Mart MF, Cunningham C (2020). Delirium. Nat Rev Dis Primers.

[38] van Sinderen K, Schwarte LA, Schober P (2020). Diagnostic criteria of postoperative cognitive dysfunction: a focused systematic review. Anesthesiol Res Pract.

[39] Liu J, Huang K, Zhu B, Zhou B, Ahmad Harb AK, Liu L, Wu X (2021). Neuropsychological tests in post-operative cognitive dysfunction: methods and applications. Front Psychol.

[40] Wang BR, Zheng HF, Xu C, Sun Y, Zhang YD, Shi JQ (2019). Comparative diagnostic accuracy of ACE-III and MoCA for detecting mild cognitive impairment. Neuropsychiatr Dis Treat.

[41] Senda M, Terada S, Takenoshita S (2020). Diagnostic utility of the Addenbrooke's Cognitive Examination - III (ACE-III), Mini-ACE, Mini-Mental State Examination, Montreal Cognitive Assessment, and Hasegawa Dementia Scale-Revised for detecting mild cognitive impairment and dementia. Psychogeriatrics.

[42] Takenoshita S, Terada S, Yoshida H (2019). Validation of Addenbrooke's cognitive examination III for detecting mild cognitive impairment and dementia in Japan. BMC Geriatr.

[43] Li X, Yang L, Yin J, Yu N, Ye F (2019). Validation study of the Chinese version of Addenbrooke's cognitive examination III for diagnosing mild cognitive impairment and mild dementia. J Clin Neurol.

[44] Zhang Y, Shan GJ, Zhang YX (2018). Propofol compared with sevoflurane general anaesthesia is associated with decreased delayed neurocognitive recovery in older adults. Br J Anaesth.

[45] Onerup A, Li Y, Afshari K (2024). Long-term results of a short-term home-based pre- and postoperative exercise intervention on physical recovery after colorectal cancer surgery (PHYSSURG-C): a randomized clinical trial. Colorectal Dis.

[46] Hameed D, Bains SS, Dubin JA (2023). Timing matters: optimizing the timeframe for preoperative weight loss to mitigate postoperative infection risks in total knee arthroplasty. J Arthroplasty.

